The article "Electroencephalogram Image under Complex Domain Analysis Algorithm to Analyze Neurological Status Epilepticus and Poor Prognostic Factors of Children" was retracted in 2023. Reasons: signs of a paper mill; suspected computer-generated content; unreliable results or conclusions; concerns about the data.

# Electroencephalogram Image under Complex Domain Analysis Algorithm to Analyze Neurological Status Epilepticus and Poor Prognostic Factors of Children

**DOI:** 10.1155/2021/3109061

**Published:** 2021-12-15

**Authors:** Jiyong Gao, Na Dai, Zhigang Liu, Dehong Chen, Junqing Zhen, Jin Wang

**Affiliations:** Department of Pediatrics, Jinan Maternity and Child Care Hospital, Jinan 250001, Shandong, China

## Abstract

This study was to adopt the electroencephalogram (EEG) image to analyze the neurological status epilepticus (SE) and adverse prognostic factors of children using the complex domain analysis algorithm, aiming at providing a theoretical basis for the clinical treatment of children with SE. 24-hour EEG was adopted to diagnose 197 children with SE. The patients were divided into an experimental group (100 cases) and a control group (97 cases) using a random number table method. The EEGs of children in the experimental group were analyzed using the compound domain analysis algorithm, and those in the control group were diagnosed by a professional doctor. The indicators of children in two groups were compared to analyze the effect of the compound domain analysis algorithm in diagnosing diseases through EEG. The prognostic scores of 197 children were scored one month after they were diagnosed, treated, and discharged, and the adverse prognostic factors were analyzed. As a result, EEG can accurately and effectively analyze the brain diseases in children. The sensitivity and specificity of the complex domain analysis algorithm for the detection of epilepsy EEG were much higher than those of the EEG automatic detection algorithm based on time-domain waveform similarity and the EEG automatic detection algorithm based on convolutional neural network (CNN), and the average running time was opposite, showing obvious difference (*P* < 0.05).The average accuracy, sensitivity, and specificity of children in the experimental group were 96.11%, 97.10%, and 95.19%, respectively; and those in the control group were 88.83%, 90.14%, and 87.82%, respectively, so there was an obvious difference in accuracy between two groups (*P* < 0.05). There were 57 cases with good prognosis and 140 cases with poor prognosis; there were 70 males with good prognosis and 19 poor prognoses and 69 women with good prognosis and 19 poor prognoses. Among 121 patients with infections, 84 cases had good prognosis and 37 cases had poor prognosis; 39 cases of irregular medication had good prognosis in 31 cases and a poor prognosis in 8 cases; and 37 cases had no obvious cause, including 25 cases with good prognosis and 12 cases with poor prognosis. In short, the EEG diagnosis and treatment effect of the compound domain analysis algorithm were better than those of professional doctors; the gender of the patient had no effect on the poor prognosis, and the pathogenic factors had an impact on the poor prognosis of the patient.

## 1. Introduction

Children's neurological epilepsy, no gender specificity, will have headaches and dizziness in the early stage of onset [1] and will be accompanied by numbness, panic, and fear. In addition, foaming at the mouth, twitching, turning up eyes, incontinence, confusion, unclear speech, and other symptoms occurred during the attack [2]. Children's neurological epilepsy disease is the damage of brain neurons, leading to abnormal discharge, causing the disease to attack. Status epilepticus (SE) is a common critical illness in neurology and the most severe form of epilepsy [3], with an annual incidence between 1 in 10,000 and 4 in 10,000 [4]. It means that epilepsy does not fully recover consciousness and frequently recurs between consecutive episodes [5], or the episodes last more than 30 minutes and do not stop spontaneously. If it is not treated for a long time, it can cause cell metabolism disorder, energy supply failure, and brain neuron death [6] and can cause irreversible damage to organs due to high fever or neuronal excitotoxic damage [7], resulting in substantial increase of disability and death rates. All kinds of epilepsy episodes can cause the occurrence of SE. During the onset of SE, children usually have partial disturbances in consciousness and motor function. Children with more serious illness [8] have a greater chance of cerebral edema and increased intracranial pressure. According to the presence or absence of strong skeletal muscle contraction during the onset, it is classified into convulsive SE (CSE) and nonconvulsive SE (NCSE) [9].

So far, among the auxiliary diagnosis methods of epilepsy, EEG examination is one of the most important, valuable, and convenient methods [10–12]. Generally speaking, about 80% of epilepsy patients have EEG abnormalities in the intermittent period, while only 5%–20% of epilepsy patients can be normal in the intermittent period, which can be diagnosed as epilepsy [13, 14]. The basic rhythm of brain electrical activity is composed of alpha waves of 8 to 13 weeks per second, and each nerve cell performs a rhythmic spontaneous discharge activity (consistent with the periodic depolarization of the nerve cell membrane), but its frequency is low and quite constant (10–20 cycles/sec) [15]. Therefore, the total discharge of nerve cells is dispersed in time, and the more dispersed the discharge time, the lower the shape amplitude of the total discharge, and the longer the duration [16]. Although CT and magnetic resonance imaging examinations can also help determine epileptic lesions, some epileptic lesions without morphological changes still need EEG to improve the accuracy of positioning [12].

Since the current detection model for epilepsy EEG images is still based on a single algorithm domain, the degree of mining and characterization of effective pathological information is not high, and the analysis effect is difficult to meet the requirements of clinical application. In addition, there are still problems in algorithm stability, adaptability, and generalization [17]. In this case, it is particularly urgent and necessary to seek an efficient and reliable method for analyzing epilepsy EEG signals. The target detection method based on composite domain can integrate the advantages of multiple domains and improve the detection accuracy while suppressing the cluttered background. It is suitable for the detection of salient target images such as natural scenery, biomedicine, architecture, and transportation [18]. In this study, the EEG intelligently identified by the complex domain analysis algorithm was adopted in this study to diagnose one of the SE, NCSE, so as to explore the effect of the complex domain analysis algorithm on the clinical diagnosis of NCSE. One month after NCSE diagnosis and treatment, the Glasgow prognosis score was performed on its prognosis, and the factors of poor prognosis were analyzed, so as to provide theoretical guidance for the clinical diagnosis and treatment of neurological epilepsy of children with higher quality and efficiency.

## 2. Materials and Methods

### 2.1. Research Objects and Their Grouping

197 children diagnosed with SE in the hospital from September 2017 to September 2020 were selected as the research objects, of which 93 were children with NCSE and the rest were CSE. They were all performed with the EEG monitoring. The children were younger than 14 years old and older than one year old. Among them, there were 99 male children and 98 female children. Children who did not cooperate in the later stage were excluded. A 24-hour EEG recording was performed on 197 children, and they were divided into an experimental group (100 cases) and a control group (97 cases) by random number table method. The EEG results in the experimental group were intelligently diagnosed by complex domain analysis algorithm, and those in the control group were diagnosed by professional doctors. A one-month long-term follow-up was performed on all discharged children to record the good and poor prognosis, observe related adverse factors, and perform prognostic scores. And the adverse factors of good prognosis were analyzed. The study had been approved by the ethics committee of hospital, and the children and their families had made comprehensive understanding of the entire research process and signed the informed consent forms.

The inclusion criteria were defined as follows: children with age range of 1∼14 years old, children whose diagnosis met the diagnostic criteria of SE proposed by the International Antiepilepsy Alliance, and children whose families agreed with the doctor to carry out the follow-up treatment of epilepsy.

The exclusion criteria were defined as follows: children with craniocerebral diseases and systemic diseases, children who could not receive continuous treatment, and children with incomplete clinical data and medical history information.

### 2.2. Discharge Mechanism of Epilepsy

Epilepsy attacks can cause changes in EEG, so studying the amplitude, waveform, and frequency of epilepsy EEG signals can effectively help clinically automatic detection of epilepsy. The characteristics of the EEG signal discharged during status epilepticus are shown in Figure 1.

Spike is a short wave with a time limit of 20∼80 ms, and it shows a vertical drop or rise with an amplitude of 100∼200 *μ*V. The polarity of the negative spike is upward, and the polarity of the positive spike is downward. A sharp slow wave is expressed as a sharp wave with a duration of 80∼120 ms followed by a slow wave with a duration of 500∼1000 ms. The sharp wave is a pathological wave with a time limit of 80 ms∼300 ns, and it is shaped like a triangle and rises slowly. The amplitude of the wave is generally above 200 *μ*V. The peak rhythm disorder is manifested as a spike wave, multiple spike waves, or multiple spikes and a slow composite wave; that is to say, the slow wave has a chaotic waveform in time and location, and the amplitude of the wave is up to 1000 *μ*V. Spike-slow wave, mainly slow wave, is a coincidence wave composed of one spike wave and one slow wave. Spike waves are all negative phase waves on the slow wave branch. Spiny slow wave refers to a combination of one or more continuous spike waves followed by a slow wave, which is more common in myoclonic epilepsy. Paroxysmal rhythm wave refers to a high-amplitude rhythm that suddenly appears in the original EEG and then suddenly disappears into a paroxysmal rhythm. The generator system of epilepsy-like discharge was shown in Figure 2.

### 2.3. EEG and Electroencephalograph

Human tissue cells will spontaneously continuously produce weak bioelectrical activities, generating pulsed currents. Impulsive synchronous potential differences were emitted by nerve cell groups in various regions of the cerebral cortex. It can be magnified by electroencephalography technology by one million times. Electrodes are installed on the scalp to draw out the electrical activity of the cells and amplified by the electroencephalograph to obtain a certain waveform, amplitude, frequency, and phase of the graph and curve, which is EEG. EEG is a curve with the electric potential of brain cells as the vertical axis and time as the horizontal axis. When a neuron is stimulated, the balance of the cell membrane is disrupted, highly depolarized, an action potential is generated, and the next stage of the balance of the cell membrane is destroyed. This repeated process of restoring and destroying the cell membrane constitutes a unidirectional transmission of action potentials on neurons and nerve cell membranes, generating brain electrical signals with an amplitude ranging from 10 to 100 *μ*V. The electroencephalograph is an instrument that picks up extremely weak EEG signals for amplification and trace recording, and its basic principle block diagram is shown in Figure 3.

Brain wave is a method of recording brain activity with electrophysiological indicators, and it is formed by the sum of the postsynaptic potentials that occur in synchronization with neurons during brain activity. The postsynaptic potential derived from the dendrites at the top of the pyramidal cells is a spontaneous and rhythmic neural electrical activity with a frequency range of 1∼30 HZ. It can be divided into four wavebands, which are delta (*δ*) wave, theta (*θ*) wave, alpha (*α*) wave, and beta (*β*) wave.  Figure 4 shows the *δ* wave with a frequency of 1∼3 Hz and an amplitude of 20∼200 pV. Generally, this kind of wave can be recorded in the parietal lobe when people are in infancy or immature intellectual development, and adults are in extreme fatigue, lethargy, or anesthesia.

As given in Figure 5, the *θ* wave showed a frequency of 4∼7 Hz and an amplitude of 5∼20 *μ*V. This wave was extremely prominent in adults who were frustrated or depressed and in children with mental illness. But this wave is the main component in the EEG of teenagers (10–17 years old).

As shown in Figure 6, it was an alpha wave with a frequency of 8∼13 Hz (average number of 10 Hz) and an amplitude of 20∼100 uV. It is the basic rhythm of normal brain waves. If there is no external stimulation, its frequency is quite constant. The rhythm is most obvious when people are awake or quiet, and when they closed their eyes; when they open their eyes, receive light stimulation, or receive other stimuli, the waves disappear instantly.

As given in Figure 7, it is a *β* wave with a frequency of 14∼30 Hz and an amplitude of 100∼150 *μ*V. This wave appears when a person is nervous and emotionally excited . When a person wakes up from a nightmare, the original slow-wave rhythm can be immediately replaced by this rhythm.

### 2.4. Complex Domain Analysis Algorithm

At present, the adaptability of traditional algorithms to different classification tasks is still weak, and it is necessary to consider the construction of adaptive automatic detection algorithms. Therefore, the Fractional Fourier Transformation (FrFT) was combined with wavelet packet transform (WPT) in this study to propose a composite domain analysis algorithm.

Fourier Transform (FT) is a very commonly used frequency domain analysis method, which can clearly obtain the overall frequency distribution of the signal, but it cannot display the time when the specific frequency appears. This defect has certain drawbacks for processing nonstationary signals, so its advanced mode FrFT is usually used in the algorithm. FrFT can reveal the time and frequency components mixed in the signal at the same time and effectively capture the small changes in the local area. Its equation can be expressed as follows:

(1) $$\begin{array}{c} \text{FrFT}=\int_{-\infty }^{+\infty }x\left(l\right)H_{f}\left(l,v\right)\text{d}l, \end{array}$$

(2) $$\begin{array}{c} H_{f}\left(l,u\right)=\left[\begin{array}{cc} \sqrt{\frac{1-i\;\cot\;\theta }{2\pi }}\times \;\exp\left(\frac{l^{2}+v^{2}}{2}\cot\;\theta -i\left(l\cdot v\right)\csc\;\theta \right) & \theta \neq b\pi \\ \lambda \left(l-v\right) & \theta =2b\pi \\ \lambda \left(l+v\right) & \theta =\left(2b+1\right)\pi \end{array}\right.. \end{array}$$

Here, *f* represented the order of FrFT, *H*_*f*_(*l*, *v*) represented the sum function, *θ* referred to the angle of rotation, and *b* was any integer. Wavelet transform was a mathematical method to solve the decomposing nonstationary signals. Compared with the FT which uses a set of infinitely long trigonometric function bases for signal fitting, the wavelet transform uses a set of orthogonal and rapidly attenuating wavelet function bases for signal fitting. This kind of wavelet function basis can obtain different frequency and time positions through its scale variable and translation variable. From the perspective of signal processing, in wavelet transform, the signal can be decomposed into high-frequency and low-frequency components through a signal filter to form a binary tree structure (Figure 8).

Therefore, FrFT and WPT were combined with domain analysis, and then fuzzy entropy signal feature extraction and classification can be constructed into a composite domain analysis algorithm. The specific process can be shown in Figure 9.

It was supposed that NCSE was positive and CSE was negative. True positive (TP) indicated that the predicted result was true and the actual was true; false positive (FP) referred to the fact that the predicted value was true and the actual was false; false negative (FN) meant that the predicted value was false and the actual was true; and the true negative (TN) meant that both the predicted value and the actual were negative. In this study, accuracy was used to indicate the proportion of correct predictions, and the specific calculation method was shown in the first following equation. Sensitivity indicated the probability of detection of a positive case, which could be calculated with the second following equation. Specificity referred to the probability of a negative case to be detected out, the calculation expression of which was shown in the third following equation:

(3) $$\begin{array}{c} \text{A}=\frac{\text{TN}+\text{TP}}{\text{TN}+\text{TP}+\text{FP}+\text{FN}}, \end{array}$$

(4) $$\begin{array}{c} \text{Se}=\frac{\text{TP}}{\text{TP}+\text{FN}}, \end{array}$$

(5) $$\begin{array}{c} \text{Sp}=\frac{\text{TN}}{\text{TN}+\text{FP}}. \end{array}$$

### 2.5. Evaluation on Treatment and Efficacy

Glasgow prognosis score covered five levels: level 1: the patients died; level 2: the patients were in a vegetative state; level 3: the patients suffered from serious sequelae and had to be assisted by other people in life; level 4: the patients suffered from moderate sequelae, and their daily life and social activities can barely be maintained by oneself; and level 5: the patients were basically healthy and can study and live normally, but some minor sequelae may also occur. Level 5 was a good prognosis, and all other levels were a poor prognosis.

NCSE diagnostic criteria were given as follows: the focal or extensive sharp waves, spike waves, or spike-slow complex waves that appeared multiple times, greater than 3 Hz; when it was less than 3 Hz, the secondary standards had to be met; abnormal brain waves with continuous periodicity and rhythm greater than 1 Hz and clear frequency changes, morphological changes, or localization changes occur, and the amplitude or sharpness changes alone were not enough. The secondary criteria were described as follows. After the use of rapid antiepilepsy drugs, clinical symptoms change rapidly or normal EEG signals appeared. Only the disappearance of spike waves did not meet the above secondary criteria, and it met the above criteria and continued to change for more than 30 minutes to confirm the diagnosis.

### 2.6. Statistical Analysis

The data processing was analyzed by SPSS version 19.0 statistical software, the count data was expressed by the percentage (%). Pairwise comparison was performed by analysis of variance, and *P* < 0.05 indicated that the difference was statistically significant.

## 3. Results

### 3.1. EEG

Figures 10–12 show the abnormal wave of the EEG of three random children with epilepsy.  Figure 10 shows the EEG of the epilepsy in the temporal lobe of the child, which revealed that the average lead showed a sharp slow wave synthesis.

Figure 11 shows a bipolar lead, which illustrated that the sharp waves of F8 and T4 were facing each other and the slow wave phase was inverted.

Figure 12 shows a partial picture of the EEG of the earphone lead. The positive sharp waves were visible and the ear poles were activated.

### 3.2. Performance Analysis of Composite Domain Analysis Algorithm

In this study, we introduced the EEG automatic detection algorithm based on time-domain waveform similarity, the EEG automatic detection algorithm based on CNN, and the composite domain analysis algorithm for comparative analysis. As shown in Figure 13, the accuracy, sensitivity, specificity, and average running time of the complex domain analysis algorithm for epilepsy EEG detection were 95.15%, 93.48%, 89.73%, and 13.41 s, respectively. The EEG automatic detection algorithm based on time-domain waveform similarity showed 90.13%, 87.82%, 78.04%, and 36.18 s for the detection accuracy, sensitivity, specificity, and average running time of epilepsy EEG, respectively. The EEG automatic detection algorithm based on CNN showed 91.65%, 89.02%, 83.33%, and 24.88 s for the detection accuracy, sensitivity, specificity, and average running time of epilepsy EEG, respectively. Among them, the sensitivity and specificity of the complex domain analysis algorithm for the detection of epilepsy EEG were obviously higher than the automatic EEG detection algorithm based on time-domain waveform similarity and the EEG automatic detection algorithm based on CNN, and the differences were greatly statistical (*P* < 0.05). The average running time of the compound domain analysis algorithm for the detection of epilepsy EEG was shorter than that of the EEG automatic detection algorithm based on time-domain waveform similarity and the EEG automatic detection algorithm based on CNN, and the differences were statistically obvious (*P* < 0.05). Compared with the EEG automatic detection algorithm based on time-domain waveform similarity and the EEG automatic detection algorithm based on CNN, the accuracy of the composite domain analysis algorithm for epilepsy EEG was not significantly different (*P* > 0.05).

### 3.3. Analysis on Neurological SE Effect Using EEG Image under Complex Domain Analysis Algorithm

Among them, there were 93 children with NCSE and 104 children with CSE. 24-hour EEG recordings were performed on them. The EEG results in experimental group were diagnosed intelligently by the complex domain analysis algorithm, and those in the control group were diagnosed by professional doctors. The evaluation was performed three times to improve the accuracy of the experimental results. As shown in Figure 14, the TPs of three times in the experimental group were 89, 90, and 92, respectively; the FPs were 4, 6, and 5, respectively; the three FNs were 4, 3, and 1, respectively; and the three TNs were 100, 98, and 99, respectively. In the control group, the three TPs were 82, 85, and 84, respectively; the three FPs were 15, 11, and 12, respectively; the three FNs were 11, 8, and 9, respectively; and the three TNs were 89, 93, and 92, respectively.

Based on the above positive and negative results, the indicators of the two groups were calculated. As shown in Figure 15, the three accuracies in the experimental group were 95.94%, 95.43%, and 96.95%, respectively; the three-time sensitivities were 95.6%, 96.77%, and 98.92%, respectively; and the three specificities were 96.15%, 94.23%, and 95.19% respectively. In the control group, the three accuracies were 86.80%, 90.36%, and 89.34%, respectively; the three sensitivities were 88.7%, 91.40%, and 90.32%, respectively; and the three specificities were 85.58%, 89.42%, and 88.46%, respectively.

As revealed in Figure 16, the average accuracy, sensitivity, and specificity of the experimental group were 96.11%, 97.10%, and 95.19%, respectively, while those in the control group were 88.83%, 90.14%, and 87.82%, respectively. There was a statistically obvious difference in accuracy between the experimental group and the control group (*P* < 0.05).

### 3.4. Analysis on Adverse Prognostic Factors

197 children were scored one month after discharge, and the results are shown in Figure 17. 19 cases were followed in level 1, 31 cases were followed in level 2, 48 cases were determined as level 3, 42 cases were determined as level 4, and 57 cases were confirmed as level 5. There are 57 cases with good prognosis and 140 cases with poor prognosis.

Whether the general information of patients affected the prognosis was analyzed, and the results are given in Figure 18. According to the analysis of gender influencing factors, 70 cases of men had good prognosis and 19 cases had poor prognosis; 69 cases of women had good prognosis, and 19 cases had poor prognosis.

The triggers were analyzed, and the results are shown in Figure 19. Among 121 cases of infections, 84 cases had good prognosis and 37 cases had poor prognosis; there were 39 cases of irregular medications including 31 cases with good prognosis and 8 cases with poor prognosis; there were 37 cases without obvious cause, including 25 cases with good prognosis and 12 cases with poor prognosis.

## 4. Discussion

Children with SE should avoid strong light stimulation and noise stimulation, stay away from noisy places, and eat less spicy food [19]; avoiding infection and forming good behaviors and mentality can effectively prevent the onset of SE and also effectively prevent the exacerbation of the disease [20]. Because SE is not clinically specific [21], its diagnosis mainly depends on EEG, which was a curve with the electrical activity of brain cells as the vertical axis [22] and time as the horizontal axis. Human brain consciousness, or brain waves, is a phenomenon derived from quantum entanglement [23]. When brain waves are excited, the surrounding quantum entangles, causing other brain waves to be entangled quantum interference [24], so that the quanta produced by other people's brain waves merge with the quanta produced by us again [25], and finally assimilated back by other quanta in the brain waves of us and others. This phenomenon is called brain wave synchronization, and the process of synchronization is called brain wave communication [26]. Children with SE need to be treated in time; otherwise it will cause intellectual disability, severely cause irreversible brain damage, and even endanger the life of the child. The prognosis of children should be evaluated as soon as possible after SE clinical diagnosis and treatment, and the factors of poor prognosis should be analyzed.

In this study, a 24-hour EEG recording was performed on children with SE, and the EEG results were intelligently diagnosed by complex domain analysis algorithm and professional doctors in two groups. The indicators of the two groups were compared to analyze the effect of the complex domain analysis algorithm in diagnosing diseases through EEG. The prognosis score was performed one month after the children were diagnosed, treated, and discharged, and the adverse factors of the prognosis were analyzed. It was found that EEG can accurately and effectively analyze brain diseases in children. The 24-hour EEG was adopted to diagnose 197 children with SE. The EEGs of children in experimental group were analyzed using the compound domain analysis algorithm, and those in the control group were diagnosed by professional doctor. The evaluation was performed three times to improve the accuracy of the experimental results. The TPs of three times in the experimental group were 89, 90, and 92, respectively; the FPs were 4, 6, and 5, respectively; the three FNs were 4, 3, and 1, respectively; and the three TNs were 100, 98, and 99, respectively. In the control group, the three TPs were 82, 85, and 84, respectively; the three FPs were 15, 11, and 12, respectively; the three FNs were 11, 8, and 9, respectively; and the three TNs were 89, 93, and 92, respectively. Based on the above positive and negative results, the indicators of the two groups were calculated. As shown in Figure 12, the three accuracies in the experimental group were 95.94%, 95.43%, and 96.95%, respectively; the three-time sensitivities were 95.6%, 96.77%, and 98.92%, respectively; and the three specificities were 96.15%, 94.23%, and 95.19%, respectively. In the control group, the three accuracies were 86.80%, 90.36%, and 89.34%, respectively; the three sensitivities were 88.7%, 91.40%, and 90.32%, respectively; and the three specificities were 85.58%, 89.42%, and 88.46%, respectively. In addition, the average accuracy, sensitivity, and specificity of the experimental group were 96.11%, 97.10%, and 95.19%, respectively, while those in the control group were 88.83%, 90.14%, and 87.82%, respectively. There was a statistically obvious difference in accuracy between the experimental group and the control group (*P* < 0.05). Such results indicated that the effect of EEG under complex domain analysis algorithm is better.

The detection performance of the composite domain analysis algorithm and the previous algorithm was compared, and it was found that the sensitivity and specificity of the composite domain analysis algorithm for the detection of epilepsy EEG were much higher than those of the automatic detection algorithm based on the time-domain waveform similarity and the CNN, while the average running time was the opposite, and the differences were significant (*P* < 0.05). Such results are similar to the results of Yao et al. [27] using regularized least squares support vector machines to identify and detect epilepsy EEG signals, indicating that the composite domain analysis algorithm has a better detection effect on epilepsy EEG images and the results are reliable. One month after the diagnosis and treatment of the children, the prognosis was evaluated and the adverse prognosis factors were analyzed. Among them, 57 cases had a good prognosis and 140 cases had a poor prognosis. In view of the analysis of the factors of poor prognosis, the general information of the patient is analyzed whether it affects the prognosis. In terms of gender, the number of male children with good prognosis (70 cases) is very similar to the number of female children with good prognosis (69 cases), and there is no significant difference between them. The reason may be that there is no obvious difference in the incidence of epilepsy between men and women and there is no gender bias in case selection. The results indicate that gender does not affect the prognosis of children with epilepsy. In terms of predisposing factors, the number of cases with good prognosis (84 cases) and the number of cases with poor prognosis (37 cases) among children with infections were significantly higher than those with irregular medications. This indicates that infection caused by irregular medication may be the risk factors affecting the prognosis of children and the effect of infection caused by disease is the most obvious.

## 5. Conclusion

In this study, the complex domain analysis algorithm diagnosis of the EEG of children with SE and the diagnosis of professional doctors were performed to compare the effects of the complex domain analysis algorithm on the diagnosis of diseases. The prognostic score was performed on the children after diagnosis, treatment, and discharge; and the adverse factors of the prognosis were analyzed, so as to provide theoretical guidance for better clinical treatment of SE. The results suggested that EEG can accurately and effectively analyze brain diseases in children and the EEG of complex domain analysis algorithm was more effective than professional doctors in diagnosing and treating diseases. In addition, the gender of the patient basically had no effect on the poor prognosis, and the pathogenic factors had a greater impact on the poor prognosis of the patient.

However, there were some shortcomings for this study. The size of sample was small, which may lead to certain limitations in the experimental results. Therefore, in future experimental studies, the sample size should be expanded, and other types of algorithms should be added for comparison so as to further explore the effect of EEG image analysis of children's neurological SE based on complex domain analysis algorithm and analyze the adverse prognostic factors of SE. In short, this study provided theoretical guidance for the clinical diagnosis and treatment of SE and a series of diseases that can be diagnosed and treated by EEG.

## Figures and Tables

**Figure 1:** The characteristics of the EEG signal discharged during status epilepticus. (a) Spike wave. (b) Sharp slow wave. (c) Sharp wave. (d) Peak rhythm disorder. (e) Ratchet slow wave. (f) Forward spike. (g) Spike wave. (h) Paroxysmal rhythm wave.

**Figure 2:** The generator system of epilepsy-like discharge.

**Figure 3:** Schematic diagram of electroencephalograph.

**Figure 4:** Schematic diagram of *δ* wave.

**Figure 5:** Schematic diagram of *θ* wave.

**Figure 6:** Schematic diagram of *α* wave.

**Figure 7:** Schematic diagram of *β* wave.

**Figure 8:** The binary tree structure of two-level decomposition.

**Figure 9:** Schematic diagram of the complex domain analysis algorithm flow.

**Figure 10:** EEG in average lead epilepsy.

**Figure 11:** EEG in bipolar lead epilepsy. (a) Fp2-F8. (b) F8-T4.

**Figure 12:** EEG in earphone lead.

**Figure 13:** Performance analysis results of the complex domain analysis algorithm. Note: a1 was the complex domain analysis algorithm; a2 was the automatic EEG detection algorithm based on time-domain waveform similarity; and a3 was the EEG automatic detection algorithm based on CNN. ^*∗*^The difference was statistically obvious in contrast to a1 (*P* < 0.05). (a) A (%). (b) Se (%). (c) Sp (%). (d) Time (%).

**Figure 14:** The data graphs of positive and negative cases in the experimental group and control group. (a) First time. (b) Second time. (c) Third time.

**Figure 15:** Comparison on accuracy, specificity, and sensitivity in two groups. Note: first time (1), second time (1), and third time (1) were the data in experimental group, while first time (2), second time (2), and third time (2) were the data in control group.

**Figure 16:** Comparison on average indicators of two groups. ^*∗*^The accuracy in the experimental group was statistically different from that in the control group (*P* < 0.05).

**Figure 17:** Prognosis score results.

**Figure 18:** Analysis on relationship between adverse factors and gender. (a) The prognosis of women and (b) the prognosis of men.

**Figure 19:** Analysis on relationship between adverse factors and trigger. The prognosis of patients with (a) infections, (b) irregular medication, and (c) no obvious cause, respectively, is shown.

## Data Availability

The data used to support the findings of this study are available from the corresponding author upon request.
